# Mitofusin-2 Restrains Hepatic Stellate Cells' Proliferation via PI3K/Akt Signaling Pathway and Inhibits Liver Fibrosis in Rats

**DOI:** 10.1155/2022/6731335

**Published:** 2022-01-17

**Authors:** Zhiping Chen, Zeyu Lin, Jiandong Yu, Haifeng Zhong, Xianhua Zhuo, Changku Jia, Yunle Wan

**Affiliations:** ^1^Department of Hepatobiliary Surgery, The Sixth Affiliated Hospital, Sun Yat-Sen University, Guangzhou 510650, Guangdong Province, China; ^2^Guangdong Provincial Key Laboratory of Colorectal and Pelvic Floor Diseases, The Sixth Affiliated Hospital, Sun Yat-Sen University, Guangzhou 510650, Guangdong Province, China; ^3^Department of Hepatobiliary Surgery, Meizhou People's Hospital, Meizhou Hospital Affiliate to Sun Yat-Sen University, Meizhou 514021, Guangdong Province, China; ^4^Department of Gastrointestinal Endoscopy, The Sixth Affiliated Hospital, Sun Yat-Sen University, Guangzhou 510650, Guangdong Province, China; ^5^Department of Hepatobiliary Surgery, The Affiliated Hangzhou First People's Hospital,School of Medicine, Zhejiang University, Hangzhou 310006, Zhejiang Province, China

## Abstract

The mitochondrial GTPase mitofusin-2 (*MFN*2) gene can suppress the cell cycle and regulate cell proliferation in a number of cell types. However, its function in hepatic fibrosis remains largely unexplored. We attempted to understand the mechanism of *MFN*2 in hepatic stellate cell (HSC) proliferation and the development of hepatic fibrosis. Rat HSC-T6 HSC were cultured and transfected by adenovirus- (Ad-) *Mfn*2 or its negative control (NC) vector (Ad-green fluorescent protein (GFP)); a rat liver cirrhosis model was established via subcutaneous injection with carbon tetrachloride (CCl_4_). Seventy-two rats were randomly divided into four groups: CCl_4_, *Mfn*2, GFP, and NC. Ad-*Mfn*2 or Ad-GFP was transfected into the circulation via intravenous injection at day 1, 14, 28, 42, or 56 after the first injection of CCl_4_ in the *Mfn*2/GFP groups. Biomarkers related to HSC proliferation and the development of hepatic fibrosis were detected using western blotting, hematoxylin-eosin and Masson staining, and immunohistochemistry. In vitro, *Mfn*2 interfered specifically with platelet-derived growth factor- (PDGF-) induced signaling pathway (phosphatidylinositol 3-kinase- (PI3K-) AKT), inhibiting HSC-T6 cell activation and proliferation. During the process of hepatic fibrosis in vivo, extracellular collagen deposition and the expression of fibrosis-related proteins increased progressively, while *Mfn*2 expression decreased gradually. Upregulating *Mfn*2 expression at the early stage of fibrosis impeded the process, triggered the downregulation of type I collagen, and antagonized the formation of factors associated with liver fibrosis. *Mfn*2 suppresses HSC proliferation and activation and exhibits antifibrotic potential in early-stage hepatic fibrosis. Therefore, it may represent a significant therapeutic target for eradicating hepatic fibrosis.

## 1. Introduction

Hepatic fibrosis, characterized by necrosis and compensatory proliferation of liver cells as well as abnormal accretion of fibrous tissue, is the critical pathological feature of various chronic liver diseases and the necessary intermediate link in the occurrence of liver cirrhosis [1, 2]. The activation of hepatic stellate cells (HSC) is the cytological basis for the formation of hepatic fibrosis, while the normal morphology is in a stationary state [3]. Activated HSC synthesize large amounts of extracellular matrices (ECM); the imbalance between ECM secretion and degradation leads to collagen deposition in the liver. Further research has indicated that activated HSC release cytokines, including transforming growth factor beta (TGF-*β*) and platelet-derived growth factor (PDGF) via an autocrine mechanism, resulting in sustained activation of HSC and the development of hepatic fibrosis [3–6]. Accordingly, HSC have become a focal target in studies on hepatic fibrosis. Several researchers have attempted to inhibit HSC activation and proliferation by reducing the cytokines required during the process or by interfering with the signal transduction [7–10]. However, experiments inhibiting cell activation directly or inducing apoptosis are seldom reported.

Mitochondria are multifunctional organelles highly related to the functional state of cells and play an important role in the cell cycle, metabolism, proliferation, and apoptosis. The mitochondrial GTPase mitofusin-2 (*MFN*2) gene (aka, the hyperplasia suppressor gene) was originally identified in vascular smooth muscle cells from spontaneously hypertensive rats by Chen et al. [11]. Located on the outer mitochondrial membrane, *MFN*2 regulates mitochondrial morphology and function and plays a crucial role in mitochondrial fusion and mitochondria-mediated apoptosis [12–14]. Low expression of intracellular *MFN*2 is a necessary condition for cells entering the proliferative phase [15]. In addition, *MFN*2 performs proapoptotic and antiproliferative functions in various cell lines, including mammary, cervical, colon, hepatocellular, and lung cancer cells [16–19]. Our previous work suggested that *MFN*2 had a negative regulatory effect on HSC proliferation, but the exact mechanism remained unclear.

PDGF, which is the strongest mitogen for HSC known to date, regulates cell proliferation and division through phosphorylation by binding to the corresponding receptors on the cell membrane [5, 20, 21]. Phosphorylation of PI3K (phosphatidylinositol 3-kinase) plays a critical role in HSC activation and mitosis; specific inhibitors of PI3K can restrict PDGF-induced proliferation [22]. *MFN*2 suppresses cell proliferation by inhibiting the PI3K-AKT signaling pathway [23]. However, the correlation between *MFN*2 and PI3K-AKT signaling in hepatic fibrosis remains largely unexplored. We hypothesized that *MFN*2 plays a role in antiproliferation via the PI3K-AKT signaling pathway during the process of hepatic fibrosis. Here, we used a recombinant adenovirus (Ad) vector for transfecting *Mfn*2 into HSC-T6 cells, a rat HSC line, to evaluate the effect of *Mfn*2 on proliferation. We also investigated the mechanism of *Mfn*2-regulated antiproliferation effects on HSC-T6 cells in vitro. Furthermore, Wistar rats were transfected to reveal the role of *Mfn*2 in hepatic fibrosis.

The aim of this article is to study the antifibrotic potential of *Mfn*2, as well as its role in the cell cycle of HSC, which is seldom reported in the existing literature. *Mfn*2 probably provides new therapeutic methods for hepatic fibrosis in the near future.

## 2. Materials and Methods

### 2.1. Cell Lines, Cell Culture, and Treatment

HSC-T6 HSC were obtained from the Chinese Academy of Science Center for Excellence in Molecular Cell Science. The cells were cultured in growth medium consisting of Dulbecco's modified Eagle's medium (DMEM; Gibco Life Technologies, Carlsbad, CA, USA) containing 4.5 g/L glucose, 5000 IU/L penicillin, 5 mg/L streptomycin, and 10% fetal bovine serum (FBS; Gibco Life Technologies) in an incubator at 37°C with a humidified atmosphere of 5% CO_2_ and 95% air. For the experiments conducted under serum-free conditions, the cells were cultured in serum-free medium for 24 h. For chemokine treatment, the cells were exposed to 20 ng/mL PDGF-BB (PeproTech, Rocky Hill, NJ, USA) for 48 h.

### 2.2. Animals and Experimental Design

All experimental protocols were conducted in accordance with the Animal Research: Reporting In Vivo Experiments (ARRIVE) guidelines, and the study was approved by the Animal Care and Use Committee of Sun Yat-sen University. Adult male Wistar rats (average body weight, 200–250 g) (Laboratory Animal Center of Sun Yat-sen University, Guangdong, China) were used in the study and were given ad libitum access to food and water at room temperature (20–22°C) with a 12-h light-dark cycle. The rats were randomly divided into two groups (*n* = 24 per group): carbon tetrachloride (CCl_4_) and negative control (NC). The rats in the CCl_4_ group received subcutaneous injection of CCl_4_ at a dose of 3 mL/kg (mixed with olive oil (50% V/V)) twice a week. The NC group was treated with vehicle only (olive oil) equivalent to the CCl_4_ group. Six rats per group were randomly selected and euthanized on days 14, 28, 42, and 56 after the first injection, separately, and the livers were harvested for further study. Another 72 rats were randomly divided into four groups: CCl_4_ (*n* = 6), *Mfn*2 (CCl_4_ + Ad-*Mfn*2, *n* = 30), GFP (green fluorescent protein) (CCl_4_ + Ad-GFP, *n* = 30), and NC (*n* = 6). The *Mfn*2 and GFP groups were each randomly divided into five subgroups (*n* = 6 per subgroup). In these subgroups, Ad-*Mfn*2 or Ad-GFP was transfected into the circulation via intravenous injection on day 1, 14, 28, or 56 after the first injection of CCl_4_. All rats were sacrificed on day 70, and their livers were removed for further study.

### 2.3. Expression Vectors and Transfection

Adr-mCMV-EGFP-*Mfn*-2 (Ad-*Mfn*2) and the NC vector (Ad-GFP) were purchased from BioWit Technologies Co. Ltd. (Shenzhen, China). The Adr-mCMV-EGFP-*Mfn*-2 recombinant adenovirus vector carried the full-length *Mfn*2 gene. The HSC-T6 cells were transfected according to standard protocols. Briefly, the cells were cultured in 6-well plates, and the medium was changed every day until 70–80% confluence was achieved. The cells were transfected with adenovirus vector at multiplicity of infection (MOI) = 250 PFU (plaque-forming units) in serum-free DMEM. At 4 h after transfection, the medium was replaced with normal DMEM supplemented with 10% FBS, and the cells were cultured for 24 h. The cells were then cultured for another 24 h in medium containing 10% FBS and PDGF-BB to detect HSC-T6 cell proliferation. The transfection efficiency was ∼70% for all experimental groups. The transfection into the animal models was as follows: 1 × 10^10^ PFU Ad-*Mfn*2 or Ad-GFP was injected via the tail vein.

### 2.4. Collection of Liver Tissue

The rats were anaesthetized with 2% pelltobarbitalum natricum, and the liver tissues were obtained and cut into pieces with an average weight of 500 mg. A portion of the specimen was stored in formaldehyde for histopathological examination, and the other portion was immediately frozen at −80°C for western blotting studies.

### 2.5. Cell Proliferation

Cell proliferation capability was detected using Cell Counting Kit-8 (CCK-8, Dojindo Molecular Technologies, Kumamoto, Japan) shade selection experiments. The cells (3 × 10^3^ per well) were plated in triplicate in 96-well plates and cultured for 24 h. At 24, 48, and 72 h after transfection, 10 *μ*L CCK-8 (5 mg/mL) was added to each well, and the cells were cultured for 4 h. The absorbance was determined at 450 nm (Varioskan Flash, Thermo Fisher Scientific, Waltham, MA, USA). The experiments were repeated at least three times.

### 2.6. Western Blot Analysis and Antibodies

The HSC-T6 cells and liver tissue lysates were extracted with radio immunoprecipitation assay (RIPA) cell lysis buffer (Beyotime Biotechnology, China), and the protein concentration in the lysates was quantified using an enhanced bicinchoninic acid (BCA) protein assay kit (Thermo Fisher Scientific) with bovine serum albumin as a standard. Equal amounts of total protein extracted from the cells or liver tissues were resolved by 10% sodium dodecyl sulfate-polyacrylamide gel electrophoresis (SDS-PAGE) and transferred to polyvinylidene fluoride (PVDF) membranes (Millipore, Burlington, MA, USA) and then probed with the following anti-rat primary polyclonal antibodies: *MFN*2 (1 : 1000; Abcam, Cambridge, MA, USA), *α*-SMA (alpha smooth muscle actin) (1 : 1000; Abcam), TGF-*β*1 (1 : 1000; Cell Signaling Technology, Danvers, MA, USA), PDGFR-*β* (1 : 2500; Abcam), phosphorylated (p)-PDGFR-*β* (1 : 1000; Cell Signaling Technology), PI3K and p-PI3K (1 : 1000; Cell Signaling Technology), AKT (1 : 1000; Cell Signaling Technology), p-AKT (1 : 2500; Cell Signaling Technology), COL1 (collagen I) (1 : 500; Millipore), and GAPDH (1 : 1000; CWBiotech, Shanghai, China). The membranes were incubated at 4°C overnight. The next day, the membranes were incubated with the appropriate secondary horseradish peroxidase-conjugated secondary antibodies (1 : 10,000, Boster Biological Technology, Wuhan, China). Specific proteins were visualized using enhanced chemiluminescence (ECL, Millipore). For quantitative analysis, band density was measured and normalized to GAPDH.

### 2.7. Hematoxylin-Eosin (HE) and Masson Staining

The rat liver tissues were fixed in 10% formaldehyde and dehydrated by graded ethanol (70%, 80%, 90%, 95%, and 100%). After permeabilization with xylene, the tissues were immersed and embedded in paraffin. The paraffin blocks were cut into 4-*μ*m slices, mounted on glass slides, and stained using standard HE staining and Masson staining techniques according to previous studies [24]. Tissue damage was evaluated by observing the inflammation, cell infiltration, interstitial edema, and cell vacuolar degeneration within the liver parenchyma under a microscope. The severity of interstitial fibrosis was estimated by scanning 10 nonrepeated fields in each sample with Masson staining and graded according to the Laennec fibrosis scoring system [25].

### 2.8. Immunohistochemistry

To analyze the protein expression of p-PDGFR-*β*, *α*-SMA, and COL1 in the liver tissues, immunohistochemistry staining assays were performed as described previously. ^24^ After baking in a 60°C incubator for 1 h, tissue sections were deparaffinized in xylene, hydrated by graded ethanol, and immersed in 3% H_2_O_2_ methanol solution for 30 min to block endogenous peroxidase activity. Next, the sections were sealed with goat serum (C-0005, Bioss Antibodies, China) and incubated at room temperature for 30 min. Then, the sections were incubated in diluted primary antibodies against p-PDGFR-*β* (1 : 100), *α*-SMA (1 : 100), and COL1 (1 : 100) in a wet box at 4°C overnight. After adding the secondary antibody, the sections were incubated for 30 min at room temperature, followed by coloration with a diaminobenzidine (DAB) horseradish peroxidase color development kit (Dako, Glostrup, Denmark) for 30∼60 sec. The nucleus was counterstained with hematoxylin for 1∼1.5 min. Afterwards, the sections were differentiated by 0.1% hydrochloric acid and alcohol, colorized to blue, dehydrated, and cleared. Finally, the sections were sealed with neutral gum and examined for expression of the target proteins using an optical microscope under ×200 magnification. The mean optical density (MOD) was measured by Image-Pro Plus 6.0 image analysis software.

### 2.9. Statistical Analysis and Image Processing Software

All statistical analyses were performed using SPSS for Windows version 20.0 (SPSS, Armonk, NY, USA). The *t*-test was used for comparing two groups; multiple groups were compared using one-way analyses of variance (ANOVA). All cell culture experiments were independently performed in triplicate and the measurement data are expressed as the mean ± standard deviation (SD). *P* < 0.05 was considered statistically significant in all cases. Canvas 16 Pro and Photoshop 7.0 were used for image gathering and processing manipulations.

## 3. Results

### 3.1. HSC-T6 Cells Transfected with Ad-*Mfn*2 Constitutively Expressed *Mfn*2

Transfection efficiency was highest when the MOI value between the adenovirus and cell was 250 PFU, as we have shown previously. Compared with the untransfected cells, HSC-T6 cells transfected with Ad-*Mfn*2 or Ad-GFP emitted green fluorescence under inverted fluorescence microscopy (Figure 1(a)). We verified *MFN*2 protein expression by western blotting 48 h after transfection. *MFN*2 protein expression levels were significantly increased in the cells transfected with Ad-*Mfn*2, compared with that of the cells transfected with Ad-GFP and the normal control (*P* < 0.01) (Figure 1(b)). The findings indicate that the *Mfn*2 gene was successfully reorganized into HSC-T6 cells and expressed the corresponding protein.

### 3.2. *Mfn*2 Inhibited HSC-T6 Cell Proliferation

Adenoviral vectors bearing *Mfn*2 or GFP and PDGF were transfected into HSC-T6 cells with the aim of measuring cell proliferation. The growth density of the cell lines was observed under normal microscopy; 24 h after treatment, HSCs incubated with PDGF and PDGF + GFP had significantly increased cell growth density compared with the control group and the *Mfn*2 group (Figure 2(a)). Furthermore, automated cell counting showed that the number of HSC incubated with PDGF + *Mfn*2 was (0.7367 ± 0.05686) × 10^6^, fewer than those incubated with PDGF [(1.2967 ± 0.7024) × 10^6^] or PDGF + GFP [(1.2967 ± 0.4042) × 10^6^] (Figure 2(b)). CCK-8 assay of cell proliferation activity indicated that HSC incubated with Ad-*Mfn*2 had significantly reduced cell proliferation compared with the control group and the GFP group, while HSC incubated with PDGF exhibited significantly increased cell proliferation (Figure 2(c)). These results indicate that *Mfn*2 can restrict HSC proliferation.

### 3.3. *Mfn*2 Suppressed Fibrosis of HSC-T6 Cells via the PDGFR-*β*-PI3K-AKT Signaling Pathway

The PI3K-AKT signaling pathway is essential for PDGF-induced cell growth in vitro [26] and is responsible for upregulating COL1 expression in HSC [27]. To elucidate the molecular mechanism by which *Mfn*2 inhibits PDGF-induced HSC proliferation, the protein expression of PDGFR-*β*, PI3K, AKT, and their phosphorylated forms, as well as *α*-SMA, TGF-*β*1, and COL1, were detected by western blotting.  Figure 3 shows that PDGF led to PDGFR-*β*, PI3K, and AKT phosphorylation, and *α*-SMA, TGF-*β*1, and COL1 protein expression in the PDGF-induced cells was higher than that in the NC group. In addition, *Mfn*2 significantly reduced the PDGF-induced phosphorylation of PDGFR-*β*, PI3K, and AKT, and *α*-SMA, TGF-*β*1, and COL1 protein expression levels were significantly lower in cells overexpressing *Mfn*2 than in cells from the PDGF + GFP, PDGF, or NC groups. The PDGFR-*β*, PI3K, and AKT protein expression levels did not differ significantly among the four groups.

### 3.4. Liver Tissue Damage and Interstitial Fibrosis Gradually Deteriorated under the Influence of CCl_4_

HE staining demonstrated that there were no histological changes in NC group livers, which had normal morphology and regular lobular structure, while CCl_4_ group livers developed remarkable pathological changes such as inflammatory cell infiltration, interstitial edema, and cell vacuolar degeneration. Masson staining showed that collagen deposition and interstitial fibrosis were significantly increased in the CCl_4_ group; there was remarkable fibrosis in the portal tract. The portal and central veins were surrounded by fibrous septa, and the lobular structure was fuzzy with clearly visible false lobules (Figure 4(a)). At days 28, 42, and 56 after the first injection of CCl_4_, the Laennec fibrosis score for the CCl_4_ group was 2.67 ± 0.52, 4.50 ± 0.55, and 5.67 ± 0.52, respectively, which was significantly different compared with that in the NC group, which was 0.50 ± 0.55, 0.42 ± 0.49, and 0.33 ± 0.41 (*P* < 0.05), respectively, indicating that the severity of interstitial fibrosis was aggravated as the modeling duration increased (Figure 4(b)).

### 3.5. Protein Expression of p-PDGFR-*β*, TGF-*β*1, *α*-SMA, and COL1 Increased While *MFN*2 Decreased Gradually in the CCl_4_ Group

Western blotting indicated that, during the duration of modeling, p-PDGFR-*β*, TGF-*β*1, *α*-SMA, and COL1 protein expression increased gradually, while *MFN*2 protein expression decreased gradually in the CCl_4_ group compared with the NC group (Figure 5(a)). p-PDGFR-*β*, *α*-SMA, and COL1 protein expression was also investigated by immunohistochemical staining, which showed that expression increased gradually over time compared with the NC group (all, *P* < 0.05) and shifted from the portal area to the lobules, demonstrating that liver tissue fibrosis was aggravated in the CCl_4_ group (Figure 5(b)).

### 3.6. Upregulated *Mfn*2 Expression at the Early Stage of Hepatic Fibrosis Alleviated Tissue Damage and the Deposition of Extracellular Collagen

HE staining showed that the histological lesions were alleviated in the *Mfn*2 group compared with the CCl_4_ and GFP groups (Figure 6(a)). Consistent with pathological changes in the liver, the amount of collagen deposition was remarkably decreased in the *Mfn*2 group (Figure 6(b)). However, such effects were significantly related to actuation duration of Ad-*Mfn*2. The histological sections revealed that transfection on day 1 of the establishment of the hepatic fibrosis model led to a much lower amount of collagen deposition in the *Mfn*2 group compared with the CCl_4_ and GFP groups by the end of the experiment (*P* < 0.001). As the time of the influence of the *Mfn*2 gene decreased, the amount of collagen deposition increased gradually. Transfection after the model had been established, that is, day 56, and was followed by no difference between the amount of collagen deposition in the *Mfn*2 group and the CCl_4_ and GFP groups (*P* > 0.05) (Figure 6(c)).

### 3.7. p-PDGFR-*β*, *α*-SMA, and COL1 Expression Decreased under the Administration of *Mfn*2 in the Early Stage of Hepatic Fibrosis

As it was shown in Figure 7, Western blotting and immunohistochemical staining indicated that p-PDGFR-*β*, TGF-*β*1, *α*-SMA, and COL1 protein expression was markedly decreased and restricted in the portal area when Ad-*Mfn*2 was transfected on the first day of CCl_4_ injection in the *Mfn*2 group compared with the CCl_4_ and GFP groups (*P* < 0.05). p-PDGFR-*β*, TGF-*β*1, *α*-SMA, and COL1 expression increased gradually with the delay in Ad-*Mfn*2 transfection and shifted from the portal area to the lobules. Transfection with Ad-*Mfn*2 when the model had been established, that is, 56 days after the first injection of CCl_4_, and was followed by no difference in the expression of the above proteins between the *Mfn*2, GFP, and CCl_4_ groups (*P* > 0.05) (Figure 7).

## 4. Discussion

This study was designed to increase our understanding of the function of *Mfn*2 in HSC proliferation and in CCl_4_-induced liver fibrosis. We found that *Mfn*2 interfered specifically with PDGF-induced signaling, resulting in the inhibition of HSC proliferation. In addition, *Mfn*2 exhibited an antifibrotic effect at the early stage of fibrosis in vivo.

Liver fibrosis is a progressive pathology of tissue damage and ECM deposition within the liver parenchyma, which may develop into cirrhosis and cancerous lesions. HSC play a critical role in excessive ECM production and secretion, leading to the deposition of collagen and fibrous septum formation [28]. In the present study, HSC proliferation was significantly inhibited after *Mfn*2 transfection. HSC activation induces the release of PDGF, a highly potent HSC mitogen, which binds to PDGFR-*β*, activating Ras and sequentially propagating the stimulatory signal via the PI3K-AKT signaling pathway [29, 30]. PDGF regulates cell proliferation and division through phosphorylation by binding to the corresponding receptors on the cell membrane [5, 20, 21]. Moreover, *Mfn*2 suppresses cell proliferation by inhibiting the PI3K-AKT signaling pathway [23]. To explore the underlying mechanism of the antiproliferation effect of *Mfn*2, we detected the protein expression of PDGFR-*β*, PI3K, AKT, and their active forms. Our results indicate that *Mfn*2 treatment dramatically decreased the protein levels of p-PDGFR-*β*, p-PI3K, and p-AKT, while PDGFR-*β*, PI3K, and AKT levels were not significantly different from that in the control group. Thus, we believe that *Mfn*2 blocked the PI3K-AKT signaling pathway by preventing PDGF binding to its receptors in the cell membrane and decreasing the phosphorylation of the corresponding receptor. Interestingly, our results also show that *Mfn*2 downregulates the expression of TGF-*β*1, which stimulates ECM synthesis and inhibits its degradation [31]. However, the mechanism is unclear and remains to be addressed in further studies.

The activation of HSC and their transformation into myofibroblast-like cells (MFBLC) are the core events of hepatic fibrosis, while increased *α*-SMA expression is the hallmark of the process. The activated HSC secrete large amounts of ECM, the components of which include COL1. Accordingly, we considered the expression of p-PDGFR-*β*, *α*-SMA, and COL1 to be appropriate indicators for evaluating the severity of fibrosis, consistent with previous studies [24, 32, 33]. Our data indicate that *α*-SMA and COL1 expression were significantly decreased under the administration of *Mfn*2 compared with the GFP control group. As *Mfn*2 has antiproliferative and antifibrotic potentiality in vitro, we hypothesized that it may have a similar effect in vivo.

Hepatic fibrosis, with pathological features that include fibrous tissue hyperplasia around the portal area and central vein, destruction of the lobular structure, and regenerative nodules, is a progressive disease [34]. Consistent with this, we found that these pathological changes deteriorated gradually in the CCl_4_ group compared with the NC group. Vacuolar degeneration of the rat hepatocytes was aggravated gradually; the destruction of the lobular structure changed from fusion necrosis to bridging necrosis, and the affected range expanded as the modeling time was prolonged. ECM secretion increased, resulting in pseudolobuli formation. Liver fibrosis induced by CCl_4_ is similar to the mechanism involved in human liver fibrosis, as well as the staging of pathological changes, which are stable and reliable [35, 36]. We therefore considered the CCl_4_-induced rat hepatic fibrosis model appropriate for subsequent exploration.

Liver fibrosis, which is mainly manifested by excessive deposition of ECM such as COL1, is a common histological change in chronic liver disease [37]. The collagen content in liver protein increases significantly during liver injury, becoming an important ECM component and ultimately leading to irreversible cirrhotic changes [38, 39]. In addition, ECM synthesis greatly influences HSC proliferation and activation, resulting in the development of fibrosis [40–42]. In the present study, both western blotting and immunohistochemistry showed that p-PDGFR-*β*, *α*-SMA, and COL1 expression increased gradually and extended within the liver parenchyma in the CCl_4_ group. Conversely, the NC group had minimal expression of the previously mentioned proteins, and they were restricted to the periportal area, which may represent the normal physiological function of the liver. Accordingly, in our opinion, the expression and location of the previously mentioned proteins are of great relevance to the severity of liver fibrosis. Our data show that p-PDGFR-*β*, *α*-SMA, and COL1 expression was markedly decreased under the administration of *Mfn*2, and they were restricted around the periportal area compared to that in the GFP and CCl_4_ groups. However, this was only observed in the rats that received *Mfn*2 intervention in the early stage of liver fibrosis; as the actuation duration of CCl_4_ was prolonged, the effect of *Mfn*2 was gradually attenuated. Transfection with *Mfn*2 when the model had been established led to there being no difference in the expression of the previously mentioned proteins between the *Mfn*2 group and the CCl_4_ group. These results all suggest that the antifibrotic effect of *Mfn*2 may be related to the inhibition of HSC proliferation, which results in the downregulation of p-PDGFR-*β*, *α*-SMA, and COL1 expression.

## 5. Conclusion

To conclude, based on our findings, we have established the framework that *Mfn*2 suppresses rat HSC proliferation and activation via the PI3K-AKT pathway by directly targeting p-PDGFR-*β* in the process of fibrosis. Moreover, *Mfn*2 exhibits antifibrotic potential in the early stage of hepatic fibrosis. Hence, *Mfn*2 probably provides new therapeutic methods for hepatic fibrosis in the near future.

## Figures and Tables

**Figure 1:** HSC-T6 cells transfected with Ad-*Mfn*-2 constitutively expressed *Mfn*-2. (a) HSC-T6 transfected by Ad-*Mfn*-2 or Ad-GFP emitted green fluorescence under the observation of the inverted fluorescence microscope (magnification × 40). (b, c) The expression level of protein *Mfn*-2 in each group. ^b^*P* < 0.01, vs. control group. *Mfn*-2: mitofusin-2; HSC: hepatic stellate cell; GFP: green fluorescent protein.

**Figure 2:** *Mfn*-2 inhibits the proliferation of HSC-T6 cells. (a) HSCs incubated with PDGF and PDGF + GFP resulted in a significant increase in cell growth density compared with the control group and the *Mfn*-2 group (magnification × 40). (b) Number of HSCs of each group. (c) *Mfn*-2 inhibited cell growth as measured by the Cell Counting Kit 8 assay in HSC-T6 cell lines. ^c^*P* < 0.001 vs. control group. PDGF: platelet-derived growth factor.

**Figure 3:** *Mfn*-2 suppresses fibrosis of HSC-T6 cells via PDGFR-*β*/PI3K/Akt signaling pathway. (a) Protein expressions of *α*-SMA, Col-1, TGF-*β*1, and *Mfn*-2 in each group. (b) Protein expressions of PDGFR-*β*, PI3K, AKT, and their phosphorylation form in each group. ^b^*P* < 0.01, ^c^*P* < 0.001, vs. control group. *α*-SMA: alpha-smooth muscle actin; Col-1: collagen type 1; TGF-*β*1: transforming growth factor-beta 1; PDGFR-*β*: platelet-derived growth factor receptor-beta; PI3K: phosphatidylinositol 3-kinase; AKT: protein kinase B; p-: phospho-.

**Figure 4:** Liver tissue damage and interstitial fibrosis gradually deteriorated under the influence of CCl_4_. (a) HE and Masson staining of liver tissue harvested from each group at the 14^th^, 28^th^, 42^nd^ and 56^th^ day after the first injection of CCl_4_/olive oil (magnification × 100). (b) Score graded by the laennec fibrosis scoring system of each group. CCl_4_: carbon tetrachloride.

**Figure 5:** Protein expression of p-PDGFR-*β*, TGF-*β*1, *α*-SMA, and Col-1 increased while *Mfn*-2 decreased gradually under the influence of CCl_4_. (a) Protein expressions of *Mfn*-2, p-PDGFR-*β*, TGF-*β*1, *α*-SMA, and Col-1 of each group at the 14^th^, 28^th^, 42^nd^ and 56^th^ days after the first injection of CCl_4_/olive oil detected by western blot. (b) Protein expressions and their location in liver tissue of p-PDGFR-*β*, *α*-SMA, and Col-1 of each group detected by immunohistochemical staining (magnification × 200).

**Figure 6:** Upregulation of the expression of *Mfn*-2 at early stage of hepatic fibrosis alleviated tissue damage and the deposition of extracellular collagen. (a, b) The histological lesions and the amount of collagen depositions were alleviated under the administration of *Mfn*-2, shown by HE and Masson staining. Such effects were significantly related to actuation duration of Ad-*Mfn*-2 (magnification × 100). (c) Score graded by the Laennec fibrosis scoring system of each group. ^c^*P* < 0.001, vs. control group.

**Figure 7:** The expressions of p-PDGFR-*β*, *α*-SMA, and Col-1 decreased under the administration of *Mfn*-2 at early stage of hepatic fibrosis. (a) Western blot showed that the protein expressions of p-PDGFR-*β*, TGF-*β*1, *α*-SMA, and Col-1 markedly decreased under the administration of *Mfn*-2, and such effects were significantly related to actuation duration of Ad-*Mfn*-2. (b–d) Immunohistochemical staining indicated that protein expressions of p-PDGFR-*β*, *α*-SMA, and Col-1 markedly decreased and restricted in portal area under the administration of *Mfn*-2 (magnification × 200).

## Data Availability

Data sharing is not applicable to this article as no datasets were generated or analysed during the current study.
